# Mechanism of Gegen Qinlian Decoction Regulating ABTB1 Expression in Colorectal Cancer Metastasis Based on PI3K/AKT/FOXO1 Pathway

**DOI:** 10.1155/2022/8131531

**Published:** 2022-01-24

**Authors:** Feng Li, Lili Chen, Jinzhou Zheng, Jianfeng Yang, Xiaoyun Song, Yu Wang, Xiqiu Zhou

**Affiliations:** Department of General Surgery, Pudong Branch, Longhua Hospital Affiliated to Shanghai University of Traditional Chinese Medicine, Shanghai 200126, China

## Abstract

It was to investigate the role of Gegen Qinlian decoction (GQD) in the regulation of ABTB1 gene based on PI3K/AKT/FOXO1 signaling pathway in colorectal cancer (CRC) metastasis. In this study, 10 cases of the CRC mouse model were established by inoculating CT26 cells into the spleen of mice, which were divided into the experimental group and the control group, 5 cases in each group; the control group was intragastrically administered with normal saline 0.3 mL/d, and the experimental group was intragastrically administered with GQD 0.2 mL/d at a ratio of 0.2 g medicinal materials/10 g for 10 days and sacrificed, and pathological sections were made. The expression density of signaling pathway PI3K/AKT/FOXO1 as well as gene ABTB1 was detected in the sections of the two groups, and the mechanism of action of this gene in the two groups of mice was studied. It was found that the densities of p-PI3K, p-AKT, and p-FOXO1 in the experimental group of mice were 26.55 g/cm^3^, 70.2 g/cm^3^, and 24.36 g/cm^3^, respectively, which were significantly increased compared with the control group, *P* < 0.05; the density of ABTB1 was 35.4 g/cm^3^, which was significantly increased compared with the control group, *P* < 0.05; the proliferation and migration ability of CRC cells in the experimental group were significantly decreased, *P* < 0.05. GQD can promote the expression of ABTB1 by activating the PI3K/AKT/FOXO1 signaling pathway, in order to inhibit the proliferation and growth ability of CRC cells.

## 1. Introduction

Colorectal cancer (CRC) is a common malignant tumor in the gastrointestinal tract. Globally, the incidence of CRC in males and females ranks the third and second most common malignant tumors, respectively, and its incidence is increasing to varying degrees in most countries in the world [1]. China belongs to a low-incidence area in the world. In recent years, with the continuous improvement of people's living standards and changes in dietary habits, the incidence of CRC in China has shown a significant increase in many areas [2]. The disease is more common in middle-aged men, most common between 40 and 70 years of age, with an incidence of about 2 : 1 in men and women. It can occur in any part of the colon or rectum, with the rectum and sigmoid colon being the most common, followed by the cecum, ascending colon, descending colon, and transverse colon [3]. It can be diagnosed by clinical manifestations, X-ray barium enema, or fiberoptic colonoscopy. Pathology shows adenocarcinoma, and a few are squamous cell carcinoma and mucinous carcinoma. The modes of CRC metastasis are lymphatic metastasis, blood metastasis, and direct spread, which account for the fourth most common malignant tumor and fatal factor, and recurrence and metastasis are the main causes of death in CRC patients [4, 5]. Early detection, early diagnosis, and radical surgery are the key to treatment. Although the 5-year survival rate of early CRC is high after operation, the long-term survival rate and prognosis of advanced CRC are still poor [6]. How to improve the therapeutic effect and survival rate of CRC has been the goal of scientists' research.

Gegen Qinlian decoction (GQD) is a classic prescription for the treatment of damp-heat syndrome in *Treatise on Cold-Attack* [7], with the effect of relieving superficies and clearing interior, governing the treatment of body heat, dry mouth, asthma and sweating, red tongue, yellow tongue fur, fast pulse rate, and intermittent stop [8]. Its clinical application has reached more than 2,000 years, the formula contains four kinds of medicinal materials of Gegen (15 g), Zhigancao (6 g), baical skullcap root (9 g), and Huanglian (9 g), which can be used with eight liters of water, first boiling Gegen, remaining six liters of water, and then other herbs are added, and they all are boiled to two liters, filtration to remove dregs, and airing soup until warm [9, 10]. GQD is mainly used for the treatment of type 2 diabetes and ulcerative colitis (UC). Studies showed that PI3K/AKT/FOXO1 signaling pathway is closely related to tumor cell growth, proliferation, survival, apoptosis, metabolism, angiogenesis, invasion and metastasis, tumor resistance, and tumor immune escape [11, 12]. However, in CRC, there are few reports on the gene regulation of ABTB1 (broad complex, tramtrack and bric a brac/poxviruses and zinc finger, BTB/POZ) by GQD based on PI3K/AKT/FOXO1 signaling pathway. It was found that GQD based on PI3K/AKT/FOXO1 signaling pathway plays an important role in the regulation of ABTB1 gene in rectal cancer metastasis [13]. Therefore, in this study, CT26 cells in logarithmic growth phase were inoculated into the spleen of BLACK/C mice to establish a colorectal cancer mouse model. The effect of GQD on the expression of ABTB1 by activating the PI3K/AKT/FOXO1 signaling pathway was studied, which provided certain experimental data for the therapeutic effect of ABTB1 gene in colorectal cancer and new research directions for the treatment of colorectal cancer.

## 2. Materials and Methods

### 2.1. Experimental Materials

In this study, the test animals were mice of BLACK/C strain provided by the Experimental Animal Center, with the number of 10 mice (F: M = 1 : 1) and body weight of 180-220 g. The experiment was completed in the Experimental Animal Center and the Pathology Laboratory. After the completion of animal experiment, the professional personnel restored the original appearance of animal carcass (skin suture, etc.), and the institution recognized by the environmental protection department performed harmless treatment such as incineration.

### 2.2. Instruments, Equipment, and Main Reagents

Table 1 is the instruments, equipment, and main reagents required during the experiment.

According to the animal mouse model, this study selected the most suitable and most used instruments and equipment in clinical practice in recent years, which was conducive to our experimental operation and results closer to clinical practice, and laid a good foundation for the clinical application and promotion of this study in the future.

### 2.3. Model Preparation and Experimental Method

Ten black/C mice were divided into two groups according to the random number table: control group and experimental group, with five mice in each group. In both groups, CT26 cells in the logarithmic growth phase were inoculated into the spleen to establish a mouse model of CRC. Mice in the control group: 0.3 mL of normal saline was intragastrically administered per day; mice in the experimental group: 0.2 mL of GQD was intragastrically administered per day at a ratio of 0.2 g of medicinal materials/10 g; both groups were intragastrically administered once a day for 10 days and sacrificed and pathological sections were made. Enzyme-linked immunosorbent assay kit was used for both groups of sections (preparation method: known antigens or antibodies were adsorbed on the surface of solid phase carrier (i.e. polystyrene microreaction plate), so that the enzyme-labeled antigen-antibody reaction was performed here. The free components in the liquid phase were removed by washing method). The expression of PI3K/AKT/FOXO1 signaling pathway was detected, and the expression of the ABTB1 gene was also detected by real-time quantitative PCR (extraction and quality detection of total RNA⟶synthesis of cDNA by reverse transcription reaction⟶PCR reaction⟶result analysis) Finally, the rectal cancer cells in the two groups of mice were subjected to scratch assay and transwell assay (steps: preparation of transwell chamber⟶preparation of cell suspension⟶inoculation of cells⟶statistics of results) to observe the expression of p-PI3K, p-AKT, p-FOXO1, and ABTB1 in mice.

### 2.4. Statistical Treatment

All data were statistically analyzed by SPSS17.0 software package. The measurement data of each group were expressed by mean ± standard deviation, the expression level of ABTB1 was compared by *t*-test, and the mean of two samples was compared by independent sample *t*-test. The positive rates of p-PI3K, p-AKT, and p-FOXO1were tested by chi-square test and Fisher's exact probability method. When *P* < 0.05, the difference was statistically significant.

## 3. Results

### 3.1. General Performance of Mice

After mice were inoculated with CT26 cells in the spleen, the anorectal temperature measured within 2 days increased to a certain extent, ranging from 37.6°C to 38.0°C, with fluffy hair, crouching and laziness, and loss of appetite, but no other significant changes; on the third day, the anal temperature increased to about 38.5°C, most mice lost weight, some had soft or loose stools, and some had mucopurulent bloody stools. Four days after given GQD by gavage, the anal temperature of experimental group began to decrease, the temperature fluctuated to around 37.8°C, and the symptoms of loose stools, hematochezia, loss of appetite, and sluggish movement were gradually relieved; most of the symptoms of mice in the control group given normal saline by gavage were not significantly relieved, of which one died on the 7th day.

### 3.2. Anatomical Observation of Mice

Almost all black/C mice showed diffuse intestinal mucosal congestion and edema, with a large amount of mucus and fibrin exudation, and some mice had small bleeding spots locally in the intestine. These lesions were obvious in sigmoid colon and rectum, and even more cauliflower-like, protruding into the intestinal cavity, with surface ulceration, bleeding, and necrosis, and the intestinal canal of the control group was more serious than that of the experimental group (Figure 1).

### 3.3. Expression of PI3K, AKT, and FOXO1 in CRC Mouse Model Tissues

PI3K and FOXO1 were mainly expressed in cytoplasm and cell membrane, and AKT was mainly expressed in nucleus. After CT26 cells were inoculated into the spleen of mice to establish colorectal cancer mouse model, the positive rates of PI3K, FOXO1, and AKT in CRC tissues were 60% (6/10), 50% (5/10), and 80% (8/10), respectively, as shown in Figures 2 and 3.

By observing Figures 2 and 3, it was found that PI3K, AKT,and FOXO1 were expressed in colorectal cancer tissues, which was of great significance for clinical diagnosis and treatment.

### 3.4. Relationship between PI3K, AKT, FOXO1, and ABTB1 Expression and Clinicopathological Features in CRC Tissues

The relationship between expression genes and clinicopathological parameters in colorectal cancer tissues is shown in Figures 4–7.

By observing Figures 4–7, it was found that the expressions of PI3K, AKT, FOXO1, and ABTB1 in colon were 40%, 70%, 40%, and 6.35, respectively, and those in rectum were 60%, 60%, 30%, and 7.51, respectively. Their expressions in CRC tissues were not related to the tumor site, *P* > 0.05, and there was no statistical significance. The expression of PI3K, AKT, FOXO1, and ABTB1 under the plasma membrane was 40%, 50%, 80%, and 4.25, respectively, and the expression of submerged plasma membrane was 80%, 90%, 30%, and 7.68, respectively. The expression in high/medium differentiation was 30%, 50%, 90%, and 4.36, in low/undifferentiated that were 80%, 80%, 30%, and 10.51. The expressions without lymph node metastasis were 30%, 70%, 70%, and 4.34, respectively, and those with lymph node metastasis were 70%, 80%, 20%, and 8.71, respectively. Their expression was related to the depth of tumor invasion, differentiation, and lymph node metastasis, *P* < 0.05, and the difference was statistically significant.

### 3.5. Expression Levels of P-PI3K, P-AKT, P-FOXO1, and ABTB1 in Mice

After the scratch test and transwell test of rectal cancer cells in mice of the two groups, the expression levels of p-PI3K, p-AKT, p-FOXO1, and ABTB1 and the proliferation and migration ability of colorectal cancer cells in mice were determined (Figures 8 and 9).

By observing Figures 8 and 9, it was found that after scratch test and transwell test, the densities of p-PI3K, p-AKT, and p-FOXO1 in the experimental group were 26.55 g/cm^3^, 70.2 g/cm^3^, and 24.36 g/cm^3^, respectively, which were significantly higher than those in the control group (*P* < 0.05); the density of ABTB1 was 35.4 g/cm^3^, which was significantly higher than that in the control group (*P* < 0.05), the proliferation and migration ability of CRC in the experimental group were significantly decreased (*P* < 0.05), and the differences were statistically significant.

## 4. Discussion

The occurrence and development of CRC are related to gene regulation. More and more studies have shown that ABTB1 is closely related to the occurrence, development, and metastasis of tumors and is a potential tumor suppressor gene [14]. It was reported in the literature that GQD can successfully express ABTB1 by activating PI3K/AKT/FOXO1 signaling pathway and inhibit the proliferation and growth ability of CRC cells, which is consistent with the results of this study [15]. In this experiment, the levels of P-PI3K/PI3K, P-AKT/AKT, and P-FoxO1/FoxO1 in the experimental group were higher than those in the control group; the positive expression rate of FoxO1 in CRC was 50%, and its expression was significantly correlated with the depth of tumor invasion, differentiation, and lymph node metastasis, which could provide some reference indicators for the occurrence and development of CRC in clinical practice.

Phosphatidylinositol 3-kinase (PI3K), an intracellular phosphatidylinositol kinase discovered by Sugimoto et al. in 1984, has lipokinase activity and protein kinase activity and is responsible for the transduction of stimulating signals such as growth factors from the cell membrane to the cytoplasm [16, 17]. The results of this study showed that the positive expression rate of PI3K in CRC was 60%, and the expression of PI3K was significantly correlated with the depth of tumor invasion, differentiation, and lymph node metastasis. Relevant literature has pointed out that activation of AKT (p-AKT) is key to the role of PI3K/AKT signaling pathway [18, 19]. Lin et al. (2017) [20] reported that p-AKT was significantly higher in CRC than in adenoma, and p-AKT was significantly correlated with the stage of CRC and the level of preoperative serum carcinoembryonic antigen (CEA). The positive rate of AKT in CRC was 80%, and the expression of AKT was significantly correlated with the depth of tumor invasion, differentiation, and lymph node metastasis, which can be used as a reference index to assess the occurrence and development of CRC in clinical practice.

Relevant studies suggested that PI3K/AKT/FOXO1 signaling pathway is widely present in various tumor cells, and activation of this pathway can inhibit apoptosis and promote cell cycle progression, thereby promoting cell growth and proliferation, while participating in tumor angiogenesis, playing an important role in tumor formation, and participating in tumor invasion and metastasis [21, 22]. GQD can successfully express ABTB1 and inhibit the proliferation and growth of tumor cells by positively regulating this signaling pathway. In this study, it was found that GQD can make the ABTB1 expression in CRC positively correlated with the expression of PI3K, p-AKT, and FOXO1, which were involved in the development of CRC while inhibiting the proliferation and metastasis of CRC.

In summary, the combined detection of PI3K, p-AKT, FOXO1, and ABTB1 expression levels can understand its clinical significance, which may play an important role in the early diagnosis of CRC, judging the malignant degree of CRC, estimating the stage of CRC, and judging the prognosis. Understanding the mechanism of occurrence and development of CRC and formulating reasonable therapeutic measures for CRC patients can also provide a theoretical basis for CRC target therapy, which has very important clinical significance.

## 5. Conclusion

In this study, a mouse model of CRC was established to explore the regulation of GQD on ABTB1 gene expression by activating the PI3K/AKT/FOXO1 signaling pathway, and it was found that compared with the control group, the expressions of p-PI3K, p-AKT, p-FOXO1, and ABTB1 in the experimental group were significantly increased, *P* < 0.05; the expressions of PI3K, AKT, FOXO1, and ABTB1 were related to the depth of tumor invasion, differentiation, and lymph node metastasis, *P* < 0.05, and the proliferation and migration ability of CRC cells in the experimental group were significantly decreased, *P* < 0.05. GQD can promote the expression of ABTB1 by activating the PI3K/AKT/FOXO1 signaling pathway, in order to inhibit the proliferation and growth ability of CRC cells. This study provides some experimental data for the therapeutic role of ABTB1 gene in CRC, but also provides a new research direction for its treatment. However, due to the relatively small sample size in this study, the experimental results need to be verified by more clinical trials.

## Figures and Tables

**Figure 1:** Anatomical images of intestinal canals in mice (marked as lesion site).

**Figure 2:** Expression in CRC tissues ((a)–(c) are PI3K, AKT, and FOXO1 (SP × 200), respectively).

**Figure 3:** Expression rate of PI3K, AKT, and FOXO1 in CRC tissues.

**Figure 4:** Expression levels of PI3K, AKT, FOXO1, and ABTB1 in different tumor sites.

**Figure 5:** Expression levels of PI3K, AKT, FOXO1, and ABTB1 in different infiltration depths.

**Figure 6:** Expression levels of PI3K, AKT, FOXO1, and ABTB1 in different differentiation degrees.

**Figure 7:** Expression levels of PI3K, AKT, FOXO1, and ABTB1 in patients with and without lymph node metastasis.

**Figure 8:** Density of p-PI3K, p-AKT, p-FOXO1, and ABTB1 in mice.

**Figure 9:** OD value of proliferation and migration of colorectal cancer cells in mice.

**Table 1:** Instruments, equipment, and main reagents.

Name	Specification	Company
Inverted microscope	DM-IRB type	LEICA, Germany
Transmission electron microscope	JEOE type	Japan
Enzyme-linked immunosorbent assay kit		Shanghai Tongwei industrial Co., Ltd.
ABI 7500 Fluorescence quantitative PCR system		Applied Biosystems (ABI), USA
PCR instrument		Bio-Rad Company, USA

## Data Availability

The data used to support the findings of this study are included within the article.
